This article has been retracted.

# Biosynthesis-Based Al_2_O_3_ Nanofiller from *Cymbopogon citratus* Leaf/Jute/Hemp/Epoxy-Based Hybrid Composites with Superior Mechanical Properties

**DOI:** 10.1155/2023/9299658

**Published:** 2023-04-20

**Authors:** L. Natrayan, Yenda Srinivasa Rao, Puthalapattu Reddy Prasad, Kul Bhaskar, Pravin P. Patil, Dereje Bayisa Abdeta

**Affiliations:** ^1^Department of Mechanical Engineering, Saveetha School of Engineering, SIMATS, Chennai, Tamil Nadu 602105, India; ^2^Department of Mechanical Engineering, Sri Sivani College of Engineering, Srikakulam, Andhra Pradesh, India; ^3^Department of Chemistry, Institute of Aeronautical Engineering, Dundigal, Hyderabad 500043, India; ^4^Department of Botany, Government Degree College Sukrauli, Kushinagar, Uttar Pradesh, India; ^5^Department of Mechanical Engineering, Graphic Era Deemed to be University, Bell Road, Clement Town 248002, Dehradun, Uttarakhand, India; ^6^Department of Civil Engineering, Ambo University, Ambo, Ethiopia

## Abstract

Metallic nanoparticles (NPs) manufactured by ecofriendly strategies have also received much interest because of their elastic scattering properties and performance in nanomaterials. Aluminium oxide nanomaterials stand out among nanomaterials due to their tremendous uses in ceramic products, fabrics, therapeutic agents, catalyst supports, sewage sludge, and biosensors. The current paper investigates the effect of the nanoparticle composition and layer sequential on the mechanical characteristics of jute (J)-hemp (H) incorporated with an aluminium oxide polymer composite. NaOH is used to change the physical aspects of both plant fibres. A total of 20 specimens were tested with varying stacking sequences and padding weight ratios. Mechanical properties like a nanocomposite's tension, bending, and ILSS was measured. Stacked series and flowability substantially impact the nanocomposite. The Group 3 nanocomposite with 2% Al_2_O_3_ has the highest tensile strength, 54.28% of the Group 1 and 2 combinations. The stack series significantly influences the material properties of nanomaterials. Because of the alternating layers of natural fabrics, Group 4 specimens have the maximum flexural strength. Group 3 composite materials have the highest ILSS because they have hemp on the outermost surface. It has been discovered that Group 4 material with a 2% Al_2_O_3_ concentration is possibly the most substantial material. The existence of Al_2_O_3_ nanoparticles in the green synthesis was confirmed by XRD analysis.

## 1. Introduction

With the advancement of the technological world, the demand for breathable, excellent mechanical properties and low-cost materials grows daily. Comprehensive studies in lightweight materials are driven by the growth of slightly elevated components [1]. As a result, scientists are interested in developing new laminates with various types of fibres using polymer composite materials. Organic fibres' appealing characteristics, like minimal price, ease of access, low toxicity, and biocompatibility, encourage developers to use them as reassurance besides substituting a few artificial reinforcing materials in composite materials [2]. Nowadays, polymer nanocomposites have a broad array of applications in many fields, including the aircraft industry, amicable, automotive, and security apparatus, due to their excellent properties such as certain rigidity and high modulus as chemical stability. Fibre-reinforced polymers can be fabricated in massive amounts and seem harder, softer, and much more feasible than traditional structural steel [3]. The majority of sections in the automobile industry have been decided to be reinforced with concrete [4]. On the other hand, automakers have come to replace traditional metal with laminated composites to reduce dead load. A 25% decrease in the vehicle's weight might save billions and billions of gallons of oil. Moreover, once damaged, composites seem complex and expensive to rebuild [5]. Due to their rigidity, fortitude, heat resistance, and exceptional wear and corrosion barrier properties, epoxies and bonding agents are commonly seen as the main ingredients for fibres of polymeric materials. However, the adhesive seems to have the drawback of causing low natural rupture [6, 7]. Numerous scientists are working to improve the characteristics of polymeric materials. Overall, two techniques have recently been used to enhance fibre-based polymeric materials' stability [8]. Improving the hardenability of adhesive and the homogenization of fibrous materials inside the polymeric aircraft of polymeric materials, various types of particles in the air filler particles are being used. Throughout the last few centuries, there has already been a surge in involvement in synthetic structures. Recently, attention has turned from pure blends to hybrids containing two or more fibres or filler particles [9]. Since 2000, there seems to be a rapid growth in scientific publications on biocomposites, padded particulate matrix composites, and fibre material polymer composites.

Aside from crossbreeding to different fibres, the impact of formability on the material characteristics of biocomposites has already been extensively studied. It has been discovered that clustering series significantly influences fracture toughness [10]. Integrating low-cost natural fibres into traditional fibre composites is thought to decrease the composite's expense. Because low-density natural fibres supplant high-grade conventional fibres like glass, carbon, and kevlar, the composite's performance deteriorates [11]. In relation to performance, appropriate filler metal has been used in some cases, resulting in considerable improvements in characteristics. A detailed review was conducted to identify a proper filler metal that fits into the fibres of a matrix while also improving its effectiveness [12]. Because of their large specific surface area, filler particles are regarded as critical components for improving the physicochemical characteristics of polymer composites. The scattering, polymeric insemination, and interlayer level measure the effectiveness of a nanofiller introduced into a matrix. The nanofiller's relatively high surface region serves as an intermediary for load transfer, an additional benefit of being used [13].

Metallic nanoparticles are being discovered to still have unique applications in electrocatalysts, pottery, microelectronics, the space program, medical technology, agricultural production, circuitry, battery packs, cleaning agents, defence, biochemical detectors, photonics, textiles, as well as food preservation [14]. Even though Al_2_O_3_ NPs appear to be more stable molecularly and hydraulically than other metallic nanostructures, they have received particular attention in the composition and configuration of the most recent antimicrobials for a financially viable biomedical field [15, 16]. Many researchers have already mentioned the biocompatibility of Al_2_O_3_ ceramic. Al_2_O_3_ NPs with high purity were the first bioceramics widely utilised in clinical applications, and it was recommended that the lifespan of Al_2_O_3_ is longer than the concerned patients. Accordingly, Al_2_O_3_ NPs have been used in several branches consisting of structural ceramics and catalysis. Numerous scientists have already noted the bioactivity of Al_2_O_3_ filler [17]. Highly pure Al_2_O_3_ NPs would be the first phytocide used in medical applications, and it has been suggested that the life expectancy of Al_2_O_3_ is high. As a result, Al_2_O_3_ NPs are used in various fields, including barrier-preventing, catalyst support, fabrics, sewage sludge, and nutrient isolation. Furthermore, Al_2_O_3_ NPs have a wide range of biological devices, including biosensing, phyto, and therapeutic agents. Moreover, such synthesised paths are somewhat costly, have potential hazards, and necessitate lengthy response times, dangerous precursor chemicals, and specialised innovative equipment [18–20]. As a result, such paths harm nature. This highlights the critical need to substitute or adjust synthetic preparatory methodologies to create a viable, spotless, nontoxic, and environmentally responsible procedure using phytoremediation and other physiological reaches. This is one of the hopeful routes for NP manufacturing because it is independent of harmful chemicals and provides natural and herbal cementing agents like extracts, phytoplankton, microorganisms, microbes, sugar content, and biopolymers for Al_2_O_3_ NP stabilisation.  Figure 1 shows the applications of Al_2_O_3_ nanoparticles [21, 22].

*Cymbopogon citratus*, also called West Indian fresh mint or merely fennel, is indeed a tropical plant native to Melanesia that has been introduced to a variety of low areas. *Cymbopogon citratus* belongs to the legume family *Leguminosae* [23]. They have simple, dark green leaves that seem to have a margin of measure. The propellers are typically 18–36 feet tall. The leaves, such as those of these grass species, have concurrent vascular bundles. *Cymbopogon citratus* is native to the South Korean archipelagos. It was widely implemented in Southeast Asia in earlier centuries [24, 25]. Lemongrass has been introduced to Borneo, Latin America, and Mexico since World War I. It is becoming naturalised all across the country's tropical and subtropical regions. *Cymbopogon citratus* is commonly known as “curly” or “sereh” inside the Philippines. Its scented leaves have long been used in frying, especially for the colon's walls and cooked chicken. The leaves of this plant can be started brewing into chai, solo, or even as a seasoning in other green teas, conveying a lemony spiciness with such gentle honey and no substantial saltiness or astringency [26]. Lemongrass is recognised as a serum sample in Sri Lanka. It has been used as a plant in preparing food and for plant oils. Lemongrass is necessary for John tubers and John Akali kyung [27, 28]. Furthermore, thanks to terpenes, cineole, carnosol, luteolin, and eugenol, lemon grass oil have a high 65–85% core. To differentiate this same oil slick, geothermal liquid-liquid extraction, humidification, and refrigeration could be used. As a natural consequence of a distillate, acidic solutions make moisturisers like face creams, balms, and serums. The major constituents in such goods are fennel oil and “negros oil.” Citronellol is a component of aromatherapy, such as Cymbopogon substances, Syzygium, and Lippi bela. Mappings can be used to improve cardiovascular health in rodents through a real impact on the concentrations of chemical agents, resulting in vasodilatory [29].

Aside from being used as nanofiller in polymer composites, surface modification of natural materials enhances the material properties. Mercerization has been the most commonly used technology for fibre-reinforced passivation among the available surface treatments. It has been noted that 5% surface treatment improves the material characteristics of jute and kenaf blends [30]. The effectiveness of NaOH-processed fibres is affected by doping concentration and process conditions. There has been additional research on fibres that shows that chemical modification enhances the efficacy of biocomposites [31].

This research investigates the effect of marijuana plant crossbreeding with jute in nanocomposites. The impact of bio-based Al_2_O_3_ nanoparticles derived from *Cymbopogon citratus* is mainly studied on the blended nanostructure's effectiveness. The influence of the layer series on material characteristics is also being investigated.

## 2. Experimental Works

### 2.1. Materials

Jute and hemp are natural materials derived from the stems of their crops with a high manufacturing quantity at a minimal price. The chosen reassurance has a lower viscosity, greater dimensional stability, and excellent mechanical properties. The fibre's cellulose content impacts its load-bearing capacity, whereas its hemicellulose concentration impacts its oxidative decomposition, wettability, and anaerobic decomposition characteristics. The lignin of a fibre influences its thermostability. As a result, such fibres are commonly used in fibre-based blends. The Amman Fibre Sector in Madurai, Tamil Nadu, India, collects both materials.

### 2.2. Green Synthesis of Al_2_O_3_ Nanoparticles

Multiple approaches have been employed to concoct Al_2_O_3_ nanoparticles; even so, those have had some drawbacks, including the more excellent price of a technique and being ecofriendly, since those that generate a significant amount of polluted air inside the ecosphere due to the utilisation of solvents and related poisonous compounds. To ameliorate such disadvantages, environmental protection strategies for manufacturing Al_2_O_3_ NPs were used, which are more feasible, emit fewer emissions and are ecofriendly, enhancing the methodologies' effectiveness.

The leaves of *Cymbopogon citratus* have been gathered in the southern hills of Tamil Nadu, India. The same leaf was thoroughly rinsed under running water before the test to remove any remaining particulate matter and potential contaminants. The leaves were then collected and cut into smaller pieces. The 30 g of freshly chopped leaves were incorporated into 150 ml of double saline solution in a 250 ml volumetric flask to make the extract, after which it was simmered for 15 minutes. After evaporation, the response mixture was spun up for 15 minutes at 12,500 rpm. The solutions were filtered through a 0.5 mm filtration system and a 0.25 mm membrane filter. Eventually, the extract was filtered, acquired, stashed, and utilised as a stabilising and pairing agent [33].

Aluminium nitrate was used as a catalyst for synthesising chemicals or substances again to synthesise Al_2_O_3_ nanomaterials. In a 200 ml bottle stirrer at 40°C, 30 ml of *Cymbopogon citratus* aqueous extract has been mixed with 100 millilitres of unburned hydrocarbon solvent. The mixture solution was then microwave-irradiated, as explained by Ansari et al. Carboxylic acids discovered in *Cymbopogon citratus* leaf extract responded together via a complex formation. The abovementioned response enabled the immediate construction of an order to meet these demands for aluminium oxide nanoparticles from chemicals or substances.  Figure 2 depicts the bioformulation of Al_2_O_3_ nanoparticles.

As described earlier, Al_2_O_3_ nanomaterials have been cleansed. The element that allows has been stopped in Ml of water to eliminate such un-interacted biomolecules and potential contaminants. To summarise, the saturated solution nanoparticle has been collected by centrifugation at ambient temperature. The flocculation process was carried out three to four times to ensure optimal detachment, and the cleansed nanoparticles were dehydrated as described earlier. The finished part has been dehydrated at 150°C and calcined for 2 hours at 1200°C.

### 2.3. Composite Preparations

The biocomposite material is made using the hand layup methodology. Bidirectional jute and hemp fibres serve as strengthening phases, epoxy acts as a lattice, and biosynthesised Al_2_O_3_ serves as a filler. Jute and hemp inserts have been slashed to 150 × 150 × 3 mm mould size. The adhesive structure and the curing agent blend in a 10 : 1 weight proportion. All polymeric samples are made with a fibre content of 30% (by weight). The nanocomposite is made with 5 different stack patterns (HHHH, JHHJ, HJJH, JHJH, and JJJJ; H and J represent hemp and jute, respectively) and 4 different weight percentages of biosynthesised alumina oxide (0%, 1%, 2%, and 3%). A maximum of 20 samples have been created using the findings further shown and aluminium oxide weight proportions.  Table 1 shows the complete classification and the concentration of a blend. The composites are subjected to a 30 kg pile for the day. Subsequently, these identical reinforced specimens are cut into the specified sizes to characterise and experiment with them.

### 2.4. Mechanical Characterization

The crystalline phase and different stages of the Al_2_O_3_ NPs have been determined using XRD with CuK*α* wavelength at temperatures ranging from 20 to 80°C and a monitoring rate of 0.02°/min. Mechanical properties such as tension were carried out following ASTM 638-03, bending following ASTM D 790-03, and ILSS following ASTM D 2344.

## 3. Result and Discussion

### 3.1. XRD-Pattern Analysis of Al_2_O_3_ Nanoparticles

Figure 3 depicts the crystalline phase and the concentration of synthesised Al_2_O_3_ NPs as determined by powder x-ray diffraction. The XRD spectra reveal the distinctive diffractogram of transition stage a-alumina (Al_2_O_3_) at 2Ѳ equates (012), (108), (112), (114), (024), (118), (216), and (310) since carbonization at 1100°C, indicating that Al_2_O_3_ has been the dominant process once inclusion above 1100°C. The typical 2Ѳ peaks of biosynthesised Al_2_O_3_ nanostructures were 43.9°, 34.0°, 58.3°, 26.3°, 69.1°, 53.4°, 38.6°, and 67.4°, and the results also show that nanomaterials have a crystalline and a tetragonal structure framework. Such morals directly correspond to the intercontinental standard of information, card details 00-010-0173 of Al_2_O_3_ [34]. The average diameter of synthesised Al_2_O_3_ NPs has been approximated to be 30.5 nm.

### 3.2. Tension Behaviour

Figure 4 demonstrate the variability in tensile strength characteristics for various geometric patterns and biosynthesised Al_2_O_3_ content. Tensile behaviour increases as the percentage of biosynthesised aluminium oxide concentrations up to 2% for reinforcement of Group 5, afterwards there is a reducing trend in the tensile strength of the samples. The highest tensile strength for biocomposite Group 3, Group 4, and Group 1 is 1% Al_2_O_3_ composition. The material with jute and hemp blinking films (Group 4) is stronger than other blends. The strength of the material with 4 levels of hemp and a 2% Al_2_O_3_ composition is 48.92 MPa. The strength of the material with alternating layers of jute and hemp with 2% Al_2_O_3_ composition is 43.73 MPa, which is 76.35% higher than the strength of a four-layered hemp matrix. It can be observed that besides substituting 2 levels of hemp with 2 layers of jute and incorporating 2% Al_2_O_3_, a capacity 54% greater than that of a multihemp composite can be accomplished. As a result, the material with an interchanging stack of jute and hemp and 1% organic synthetic Al_2_O_3_ may be suggested for demanding applications with approximately 54% of the toughness of marijuana plant fibre laminates [25, 35].

Figure 5 shows the tensile modulus of biosynthesised Al_2_O_3_/jute/hemp/epoxy hybrid composites. The increased tensile strength achieved by the nanostructure could be described as follows: the reinforced framework is better suited to prolonged Al_2_O_3_. Exceptional dispersion and appropriateness benefit not just for packing between many jutes and hemp/epoxy, but also for nanoparticle electricity absorption all through brittle materials. Furthermore, 3 wt. % Al_2_O_3_ loading throughout jute/hemp/epoxy may result in primary Al_2_O_3_ aggregates causing tension force via fracture diagnosis [36, 37]. This incidence has also resulted in harmful forces applied from the interlayer to natural fabrics or emulsifiers, likely to result in material property degradation.

### 3.3. Bending Characteristics

Figure 6 shows bending strength of biosynthesised Al_2_O_3_/jute/hemp/epoxy hybrid composites. It should be mentioned that, unlike some other blends, the reinforcement of Group 4 lacks content geometry across its width. For outstanding performance, the three-point flexural test of Group 4 blends is conducted with hemp at the bottommost stack and jute fibre at the outermost layer because cannabidiol is greater in tensile stresses than jute, and the material can withstand extra flexural pile.

Figure 7 shows the flexural modulus of biosynthesised Al_2_O_3_/jute/hemp/epoxy hybrid composites. The inclusion of Al_2_O_3_ reduces the flexural strength of the majority of a hybrid composite. In contrast to the tensile strength and modulus introduced, there was no real advancement in flexible pavements with adding Al_2_O_3_. Consequently, flexural behaviours have been enhanced by 12% and 8%, respectively, once compared to a short-staffed mixture [38]. The greater flexibility and modulus seem to be caused by improved sprinkling and solubilization of Al_2_O_3_ inside the matrix material, which is consistent with the thermomechanical investigative process, resulting in more stress transfer efficiency as well as a more significant effect.

### 3.4. ILSS Behaviour

A short-beam testing procedure is used to carry out the testing. It is carried out using three flexing fittings. The method indicates that the specimen is short enough to minimise bending moment, and the fracturing is caused by interlaminar shear failure all along the flat direction between lamellae.  Figure 8 depicts the ILSS qualities for nanocomposite. The existence of robust lignocellulosic materials at the outermost surface, which is more significant in tensile stresses, results in the highest ILSS for Group 3 nanocomposite with 0% Al_2_O_3_. During experiments, it was discovered that the fracture in Group 2 nanocomposite begins to propagate from the bottom layer of jute, which is relatively weak in tensile stresses [39]. When the fracture attains the cannabidiol layer, failure mode begins since the debonding power among jute and hemp is less than the strength properties of cannabis plants [40]. This could be attributed to the fact that nanocomposite with jute at the outermost surface (Group 2) has a lower ILSS than nanocomposite with cannabis plants at the outer surface (Group 3). The results demonstrate that implementing kenaf/sisal fabric in addition to nanocrystals into epoxy has a beneficial influence on the frictional force of nanostructures and the disused framework polymers [41].

The ILSS reaction of blends is being used to evaluate whether shear behaviours exist between the substances' strands. The ILSS experiment is used on nanocomposites to assess the adhesion among strands and their resisting deformation stress at a specific point. The flexing yield strength and deflection among sheets heavily depend on stack debonding. If the load is composed of a single ply, failure between reinforcement strands results in total disaster. The ILSS experiment is used to evaluate this failure. In summary, elevated ILSS values suggest robust connective tissue between the nanofluff mixture and the reinforcement phase.

## 4. Conclusion

This study summarised the present incarnation of functionalization of Al_2_O_3_ NPs utilising *Cymbopogon citratus* vegetation in contrast to Al_2_O_3_ NPs. As a result, the scientific world must devote special attention to improving such an effective, rapid, viable, foul-smelling, reasonably priced, and ecofriendly technique for biosynthetic pathways of Al_2_O_3_ NPs using this [32] green chemical bottom-to-top approach. Furthermore, the material characteristics of a jute-hemp-biosynthesis based on Al_2_O_3_-epoxy premised polymer nanocomposites with differing stack series, and filler particles wt. % are investigated.

- The nanocomposite in Group 3 with 2% Al_2_O_3_ has the highest tensile strength, 54.28% of the Group 1 configurations. The stack series has a significant effect on the mechanical properties of nanocomposites.
- Group 4 specimens have the highest flexural strength due to the interchanging strands of natural fibres. The highest ILSS is found in composite materials with hemp at the outermost surface, i.e., Group 3. It is discovered that material concocted in Group 4 with a 2% Al_2_O_3_ concentration is perhaps the most significant.
- The typical 2Ѳ peaks of biosynthesised Al_2_O_3_ nanostructures were 43.9°, 34.0°, 58.3°, 26.3°, 69.1°, 53.4°, 38.6°, and 67.4°, and the results also show that nanomaterials have a crystalline and a tetragonal structure framework. The average diameter of synthesised Al_2_O_3_ NPs has been approximated to be 30.5 nm.

## Figures and Tables

**Figure 1:** Applications of Al_2_O_3_ nanoparticles.

**Figure 2:** Green synthesis of Al_2_O_3_ nanoparticles from *Cymbopogon citratus* leaves.

**Figure 3:** XRD-patten analysis of biosynthesis-based Al_2_O_3_ nanoparticles.

**Figure 4:** Tensile strength of biosynthesised Al_2_O_3_/jute/hemp/epoxy hybrid composites.

**Figure 5:** Tensile modulus of biosynthesised Al_2_O_3_/jute/hemp/epoxy hybrid composites.

**Figure 6:** Bending strength of biosynthesised Al_2_O_3_/jute/hemp/epoxy hybrid composites.

**Figure 7:** Flexural modulus of biosynthesised Al_2_O_3_/jute/hemp/epoxy hybrid composites.

**Figure 8:** ILSS behaviour of biosynthesised Al_2_O_3_/jute/hemp/epoxy hybrid composites.

**Table 1:** Parameter design of biosynthesised jute/hemp/epoxy composites.

Sl. no	Groups	Combinations	Weight proportions of Al_2_O_3_ (wt. %)	Symbols
1	Group 1	HHHH	0	A
2			1	B
3			2	C
4			3	D

5	Group 2	JHHJ	0	E
6			1	F
7			2	G
8			3	H

9	Group 3	HJJH	0	I
10			1	J
11			2	K
12			3	L

13	Group 4	JHJH	0	M
14			1	N
15			2	O
16			3	P

17	Group 5	JJJJJ	0	Q
18			1	R
19			2	S
20			3	T

## Data Availability

The data used to support the findings of this study are included within the article. Should further data or information be required, these are available from the corresponding author upon request.

## References

[1] Sarker F., Potluri P., Afroj S., Koncherry V., Novoselov K. S., Karim N. (2019). Ultrahigh performance of nanoengineered graphene-based natural jute fiber composites. *ACS Applied Materials and Interfaces*.

[2] Chowdary M. S., Raghavendra G., Kumar M. S. R. N., Ojha S., Boggarapu V. (2022). Influence of nano-silica on enhancing the mechanical properties of sisal/kevlar fiber reinforced polyester hybrid composites. *Silicon*.

[3] Seeniappan K., Venkatesan B., Krishnan N. N. (2022). A comparative assessment of performance and emission characteristics of a DI diesel engine fuelled with ternary blends of two higher alcohols with lemongrass oil biodiesel and diesel fuel. *Energy and Environment*.

[4] Rajeshkumar G. (2021). A comprehensive review on natural fiber/nano-clay reinforced hybrid polymeric composites: materials and technologies. *Polymer Composites*.

[5] Hasan K. M. F., Horv G., Alp T. (2020). Potential natural fiber polymeric nanobiocomposites: a review. *Polymers (Basel)*.

[6] Zhang M., Rong M., Zhang H., Rich K. F. (2003). Mechanical properties of low nano-silica. *Polymer Engineering and Science*.

[7] Habibi M. H., Fakhri F. (2017). Hydrothermal synthesis of nickel iron oxide nano-composite and application as magnetically separable photocatalyst for degradation of Solar Blue G dye. *Journal of Materials Science: Materials in Electronics*.

[8] Kim K., Mantena P. R., Daryadel S. S., Boddu V. M., Brenner M. W., Patel J. S. (2015). Dynamic Mechanical Analysis and High Strain-Rate Energy Absorption Characteristics of Vertically Aligned Carbon Nanotube Reinforced Woven Fiber-Glass Composites. *Journal of Nanomaterials*.

[9] Kaliappan A. S., Mohanamurugan S., Nagarajan P. K. (2020). Numerical investigation of sinusoidal and trapezoidal piston profiles for an IC engine. *Journal of Applied Fluid Mechanics*.

[10] Calandra P., La Parola V., Liveri V. T., Lidorikis E., Finocchi F. (2013). Composite nanoparticles. *Journal of Chemistry*.

[11] Mohammed L., Ansari M. N. M., Pua G., Jawaid M., Islam M. S. (2015). A review on natural fiber reinforced polymer composite and its applications. *International Journal of Polymer Science*.

[12] Gowda Y., Girijappa T., Rangappa S. M. (2019). Natural fibers as sustainable and renewable resource for development of eco-friendly composites. *A Comprehensive Review*.

[13] Velmurugan G., Babu K. (2020). Statistical analysis of mechanical properties of wood dust filled Jute fiber based hybrid composites under cryogenic atmosphere using Grey-Taguchi method. *Materials Research Express*.

[14] Agarwal J., Sahoo S., Mohanty S., Nayak S. K. (2019). Progress of novel techniques for lightweight automobile applications through innovative eco-friendly composite materials: a review. *Journal of Thermoplastic Composite Materials*.

[15] Mahmudi R., Poole W. J. (2009). Enhanced properties of Mg-based nano-composites reinforced with Al 2 O 3. *Materials Science and Engineering: A*.

[16] Benavente R., Pruna A., Borrell A. (2015). Fast route to obtain Al 2 O 3 -based nanocomposites employing graphene oxide: synthesis and sintering. *Materials Research Bulletin*.

[17] Cai H., Yan F., Xue Q., Liu W. (2003). Investigation of tribological properties of Al 2 O 3 -polyimide nanocomposites. *Polymer Testing*.

[18] Oh S., Lee J., Sekino T., Niihara K. (2001). Fabrication of Cu dispersed Al 2 O 3 nanocomposites using Al 2 O 3/CuO and Al 2 O 3/Cu-nitrate mixtures. *Scripta Materialia*.

[19] Ahamed H., Senthilkumar V. (2011). Consolidation behavior of mechanically alloyed aluminum based nanocomposites reinforced with nanoscale Y 2 O 3/Al 2 O 3 particles. *Materials Characterization*.

[20] Sadeghi B., Shamanian M., Ashrafizadeh F., Cavaliere P., Rizzo A. (2017). Influence of Al 2 O 3 nanoparticles on microstructure and strengthening mechanism of Al-based nanocomposites produced via spark plasma sintering. *Journal of Materials Engineering and Performance*.

[21] Sadeghi B., Cavaliere P., Perrone A., Perrone A. (2018). Effect of Al 2 O 3, SiO 2 and carbon nanotubes on the microstructural and mechanical behavior of spark plasma sintered aluminum based nanocomposites. *Particulate Science and Technology*.

[22] Dass K., Chauhan S. R., Gaur B. (2016). Study on the effects of nano particulates of sic, Al 2 o 3 and zno on the mechanical and tribological performance of epoxy based nanocomposites. *Particulate Science And Technology*.

[23] Jain S., Mehata M. S. (2017). Medicinal plant leaf extract and pure flavonoid mediated green synthesis of silver nanoparticles and their enhanced antibacterial property. *Scientific Reports*.

[24] Cai Z., Remadevi R., Al Faruque A., Setty M., Fan L. (2019). Fabrication of a cost-effective lemongrass ( cymbopogon citratus ) membrane with antibacterial activity for dye removal. *RSC Advances*.

[25] Han Lyn F., Nur Hanani Z. A. (2020). Effect of lemongrass (cymbopogon citratus ) essential oil on the properties of chitosan films for active packaging. *Journal of Packaging Technology and Research*.

[26] Natrayan L., Sundaram P. S. S., Elumalai J. (2019). Analyzing the uterine physiological with MMG signals using SVM. *International journal of pharmaceutical research*.

[27] Thangam R., Suresh V., Kannan S. (2014). Optimized extraction of polysaccharides from Cymbopogon citratus and its biological activities. *International Journal of Biological Macromolecules*.

[28] Bonferoni M. C., Sandri G., Rossi S. (2017). A novel ionic amphiphilic chitosan derivative as a stabilizer of nanoemulsions . Improvement of antimicrobial activity of Cymbopogon citratus essential oil. *Colloids and Surfaces B: Biointerfaces*.

[29] Da A., Medeiros C., Ucia M. L. (2016). Inactivation of escherichia coli, listeria monocytogenes, and salmonella enteritidis by cymbopogon citratus d c stapf essential oil in pineapple juice. *Journal of Food Protection*.

[30] Natrayan L., Kumar M. S. (2020). Influence of silicon carbide on tribological behaviour of AA2024/Al2O3/SiC/Gr hybrid metal matrix squeeze cast composite using Taguchi technique. *Materials Research Express*.

[31] Karthikeyan A., Balamurugan K., Kalpana A. (2014). The effect of sodium hydroxide treatment and fiber length on the tensile property of coir fiber-reinforced epoxy composites. *Science and Engineering of Composite Materials*.

[32] Kuppusamy P., Yusoff M. M., Govindan N. (2014). Biosynthesis of metallic nanoparticles using plant derivatives and their new avenues in pharmacological applications - an updated report. *Saudi Pharmaceutical Journal*.

[33] Meena P. R., Singh A. P., Tejavath K. K. (2020). Biosynthesis of silver nanoparticles using cucumis prophetarum aqueous leaf extract and their antibacterial and antiproliferative activity against cancer cell lines. *ACS Omega*.

[34] Archana D. P., Reddy H. N. J., Paruti B. (2022). Mechanical characterization of biocomposites reinforced with untreated and 4% NAOH-treated sisal and jute fibres. *Advances in Materials Science and Engineering*.

[35] Ahmad I., Unwin M., Cao H. (2010). Multi-walled carbon nanotubes reinforced Al 2 O 3 nanocomposites: mechanical properties and interfacial investigations. *Composites Science and Technology*.

[36] Shankar V. S., Velmurugan G., Kaliappan S. (2022). Optimization of CO 2 concentration on mortality of various stages of callosobruchus maculatus and development of controlled atmosphere storage structure for black gram grains. *Adsorption Science and Technology*.

[37] Sabarinathan P., Annamalai V. E., Vishal K. (2022). Experimental study on removal of phenol formaldehyde resin coating from the abrasive disc and preparation of abrasive disc for polishing application. *Advances in Materials Science and Engineering*.

[38] Deepak K., Reddy N. S., Naidu T. S. (2015). Thermosetting polymer and nano clay based natural fiber bio- composites. *Procedia Materials Science*.

[39] Atmakuri A., Palevicius A., Vilkauskas A., Janusas G. (2020). Review of hybrid fiber based composites with nano particles — material properties and applications. *Polymers (Basel)*.

[40] Velmurugan G., Babu K., Flavia L. I., Stephy C. S., Hariharan M. (2020). Utilization of grey Taguchi method to optimize the mechanical properties of hemp and coconut shell powder hybrid composites under liquid nitrogen conditions. *IOP Conference Series: Materials Science and Engineering*.

[41] Yasir M., Al A., Ullah Z., Ahmed W., Arshad H., Ali A. (2021). Results in Engineering Natural fiber reinforced composites: sustainable materials for emerging applications. *Results in Engineering*.

